RETRACTED

# Long non-coding RNA HOTAIR promotes UVB-induced apoptosis and inflammatory injury by up-regulation of PKR in keratinocytes

**DOI:** 10.1590/1414-431X20186896

**Published:** 2018-06-11

**Authors:** Guo Liu, Wenhao Zhang

**Affiliations:** Department of Burns and Plastic Surgery, Jining No.1 People's Hospital, Jining, Shandong, China

**Keywords:** HOTAIR, UVB-induced apoptosis, Inflammatory injury, PKR, Keratinocytes

## Abstract

Excessive exposure to ultraviolet (UV) rays can cause damage of the skin and may induce cancer, immunosuppression, photoaging, and inflammation. The long non-coding RNA (lncRNA) HOX antisense intergenic RNA (HOTAIR) is involved in multiple human biological processes. However, its role in UVB-induced keratinocyte injury is unclear. This study was performed to investigate the effects of HOTAIR in UVB-induced apoptosis and inflammatory injury in human keratinocytes (HaCaT cells). Quantitative real-time polymerase chain reaction was performed to analyze the expression levels of HOTAIR, PKR, TNF-α, and IL-6. Cell viability was measured using trypan blue exclusion method and cell apoptosis using flow cytometry and western blot. ELISA was used to measure the concentrations of TNF-α and IL-6. Western blot was used to measure the expression of PKR, apoptosis-related proteins, and PI3K/AKT and NF-κB pathway proteins. UVB induced HaCaT cell injury by inhibiting cell viability and promoting cell apoptosis and expressions of IL-6 and TNF-α. UVB also promoted the expression of HOTAIR. HOTAIR suppression increased cell viability and decreased apoptosis and expression of inflammatory factors in UVB-treated cells. HOTAIR also promoted the expression of PKR. Overexpression of HOTAIR decreased cell viability and increased cell apoptosis and expression of inflammatory factors in UVB-treated cells by upregulating PKR. Overexpression of PKR decreased cell viability and promoted cell apoptosis in UVB-treated cells. Overexpression of PKR activated PI3K/AKT and NF-κB pathways. Our findings identified an essential role of HOTAIR in promoting UVB-induced apoptosis and inflammatory injury by up-regulating PKR in keratinocytes.

## Introduction

Human skin is repeatedly exposed to chronic ultraviolet (UV) irradiation; however, excessive exposure to UV can cause either acute or chronic skin injury (1). Short-term exposure to ultraviolet B (UVB) can cause sunburn and erythema, while long-term exposure induces various cellular responses, such as inflammation, aging, and skin cancer (2,3). UV exposure induces apoptosis of keratinocytes. Additionally, insufficient repair of UV-induced DNA damage may initiate apoptosis in sunburn cells (4).

During inflammation, pro-inflammatory mediators, including cytokines, chemokines, and prostaglandins are produced, mostly by keratinocytes at the irradiated site (5). It was also found that excessive UVB irradiation increased the production of reactive oxygen species, influenced the cell metabolic pathway, and decreased the activity of superoxide dismutase (3). Therefore, it is of great importance to study the damage and regulation of UVB on skin keratinocytes for the clinical treatment of skin injury and skin cancer.

RETRACTED

Long chain non-coding RNAs (lncRNAs) are a class of non-protein coding RNAs with more than 200 nucleotides in length, and with a role in regulating protein transcriptions (6). At present, research on lncRNAs is still in the beginning stage. lncRNAs exert critical functions in adult tissue stem cells, including skin, brain, and muscle, as well as in developmental patterning and pluripotency (7). A previous study showed that lncRNA-p21 was upregulated in UVB-treated human keratinocytes (HaCaT cells) and played a significant role in cell apoptosis (8).

HOX antisense intergenic RNA (HOTAIR) is a recently discovered lncRNA that plays a critical role in gene regulation and chromatin dynamics. HOTAIR has been shown to be dysregulated in a variety of cancers (9). Rinn et al. (10) introduced HOTAIR as a spliced and polyadenylated RNA with 2158 nucleotides and 6 exons. In addition, studies showed that HOTAIR could induce the expression of TNF-α in lipopolysaccharide-induced myocardial cell inflammatory injury (11). HOTAIR is considered as a promoter of inflammatory response (12). By studying mechanisms of HOTAIR in cell injury, here, we identified a role for double-stranded RNA-dependent protein kinase (PKR) in inflammasome activation. PKR has been identified as a necessary protein kinase for the activation of one or several types of inflammasomes (13). PKR deficiency could inhibit the secretion of IL-1β, IL-18, and high mobility group box 1 (HMGB1) in *Escherichia coli*-induced peritonitis (13). PKR upregulation was shown to be related to IL-24-induced apoptosis (14). However, little is known about the effects of HOTAIR and PKR on UVB-induced keratinocyte injury. In the present study, we explored the effects of HOTAIR on UVB-induced apoptosis and pro-inflammatory response in keratinocytes and analyzed the role of PKR in the action of HOTAIR.

## Material and Methods

### Cell culture and UVB treatment

Immortalized human keratinocytes, HaCaT cells, were purchased from the Chinese Academy of Sciences (China). The cells were cultured in DMEM/F12 (Gibco, USA), supplemented with 10% fetal bovine serum at 37°C under an atmosphere of 5% CO_2_ and 95% air. HaCaT cells were plated onto culture dishes. The cells were then irradiated, covered with a thin layer of phosphate buffer saline (PBS), and exposed to UVB (30 mJ/cm^2^, 280–320 nm) for 8, 16, and 24 h from a bank of lamps (Spectronics Corp., USA) that were placed at a distance of 25 cm. The irradiance of the lamps was calculated by a calibrated photometer (Spectronics Corp.). Cells with no UVB treatment were considered as the control. The cells were supplied with fresh culture medium after exposure to UVB and incubated for subsequent studies.

RETRACTED

### Viability assay

For the viability assay, 10^5^ cells per well were plated in 24-well plates until attachment. Cells were then trypsinized and stained with trypan blue dye (Beyotime Biotechnology, China); viable cells were counted using a cell-counting chamber (Thermo Fisher Scientific, USA).

### Apoptosis assay

Flow cytometry analysis was performed to identify and quantify the apoptotic cells. The assay was done using Annexin V-FITC/PI apoptosis detection kit (Beijing Biosea Biotechnology, China) according to the protocol. The cells (10^5^ cells/well) were seeded in 6-well plates. The cells were washed twice with cold PBS and then resuspended in 195 μL binding buffer and 5 μL Annexin V-FITC solution. PI (10 μL) was added to the mixture, which was then co-incubated for 30 min at room temperature in the dark. Finally, flow cytometry (Beckman Coulter, USA) was conducted to differentiate apoptotic cells (Annexin-V positive and PI-negative) from necrotic cells (Annexin-V and PI-positive).

### siRNAs transfection

Cells transfected with si-PKR and the negative controls (NC) were synthesized by GenePharma Co. (China). Cell transfection was conducted using Lipofectamine 3000 reagent (Invitrogen, USA) following the manufacturer's protocol.

### Transfection and generation of stably transfected cell lines

Short-hairpin RNA directed against HOTAIR was ligated into the pcDNA3.1 plasmid (GenePharma, China) and was referred to as sh-HOTAIR. The sh-HOTAIR sequences were as follows: sense, 5′-GATCCGCCACATGAACGCCCAGAGATTTTCAAGAGAAATCTCTGGGCGTTCATGTGGTTTTTTG-3′, and anti-sense, 5′-AATTCAAAAAACCACATGAACGCCCAGAGATTTCTCTTGAAAATCTCTGGGCGTTCATGTGGCG-3′. The plasmid carrying non-targeting sequence was used as NC of sh-HOTAIR and was referred to as sh-NC. Plasmids overexpressing HOTAIR were ligated into the pcDNA3.1 and referred to as pc-HOTAIR. The full-length PKR sequences were constructed into pcDNA3.1 plasmids (GenePharma) to analyze the functions of PKR, and were referred to as pc-PKR. PKR siRNA was obtained from Bioneer (Daejeon Korea) with a sequence of 5′-CGUUGCUUAUGAAUGGUCU-3′. Lipofectamine 3000 reagent (Life Technologies Corporation, USA) was used for cell transfection according to the manufacturer's instructions. The stably transfected cells were selected by the culture medium containing 0.5 mg/mL G418 (Sigma-Aldrich, USA). After approximately 4 weeks, G418-resistant cell clones were established.

RETRACTED

### Enzyme-linked immunosorbent assay (ELISA)

After different treatments of HaCaT cells, the culture supernatant was collected from 24-well plates and inflammatory cytokines were quantified using specific ELISA kits for tests of TNF-α (#DTA00C) and IL-6 (#D6050) concentrations according to the protocol supplied by the manufacturer (R&D Systems, UK) and normalized to cell protein concentrations.

### Quantitative real-time polymerase chain reaction (qRT-PCR)

Total RNA was isolated from the cells using TRIzol reagent (Invitrogen) and treated with DNaseI (Promega, USA). RNA (1 µg) was reverse-transcribed in a 20 µL reaction mixture using the MultiScribe RT kit (Applied Biosystems, USA) and random hexamers or oligo(dT). The reverse transcription conditions were 10 min at 25°C, 30 min at 48°C, and 5 min at 95°C. The cDNA was amplified in a 20 µL reaction mixture. The PCR conditions were as follows: 0.4 µM of each primer, 0.2 mM deoxynucleoside triphosphate mixture (Perkin-Elmer, USA), 50 mM KCl, 10 mM Tris-HCl (pH 8.3), 1.5 mM MgCl_2_, and 1.0 U of Taq DNA polymerase (Perkin-Elmer, USA). The reaction mixtures were incubated in a thermal controller for 35 cycles (denaturation at 94°C for 45 s, annealing at 55°C for 45 s, extension at 72°C for 90 s). The specific HOTAIR primers were: forward, 5′-CAGTGGGGAACTCTGACTCG-3′; reverse, 5′-GTGCCTGGTGCTCTCTTACC-3′. The specific PKR primers were: forward, 5′-CAGAATTGACGGAAAGACTTAC GTT-3′; reverse, 5′-CATGATCAAGTTTTGCCAATGC-3′. HOTAIR levels were normalized to GAPDH: forward, 5′-GTC AACGGATTTGGTCTGTATT-3′; reverse, 5′-AGTCTTCTGGGTGGCAGTGAT-3′.

### Western blot

The proteins used for western blotting were extracted using RIPA lysis buffer (Beyotime Biotechnology) supplemented with protease inhibitors (Roche, Switzerland). The proteins were quantified using BCA™ Protein Assay Kit (Pierce, USA). Bio-Rad Bis-Tris Gel system (Hercules, USA) was used to establish western blotting system according to the manufacturer's instructions. Samples were separated by 10% SDS-PAGE and transferred to a polyvinylidene difluoride membrane (PVDF, GE Healthcare, Germany). Primary antibodies were prepared in 5% blocking buffer (5% non-fat milk in TBS-T (20 mmol/L Tris-HCl (pH 7.6), 137 mmol/L NaCl, 0.1% Tween20) at a dilution of 1:1.000. The used primary antibodies were listed as follows: Bcl-2 (ab32124), Bax (ab32503), pro-caspase-3 (ab44976), cleaved-caspase-3 (ab32042), pro-caspase-9 (ab32539), cleaved-caspase-9 (ab32539), IL-6 (ab6672), TNF-α (ab1793), PKR (ab32506), PI3K (ab86714), p-PI3K (ab182651), AKT (ab32505), p-AKT (ab131443), p65 (ab16502), p-p65 (ab86299), IκBα (ab32518), p-IκBα (ab32518), and GAPDH (ab9485, Abcam, USA). The membrane was incubated with primary antibody at 4°C overnight, followed by washing and incubation with goat anti-rabbit (ab205718) or goat anti-mouse IgG (ab6789) marked by horseradish peroxidase for 1 h at room temperature. After rinsing, the PVDF membrane carrying the blots and antibodies were transferred onto Bio-Rad ChemiDoc™ XRS system, and 200 μL Immobilon Western Chemiluminescent HRP Substrate (Millipore, USA) was added to cover the membrane surface. The signals were captured and the intensity of the bands was quantified using Image Lab™ Software (Bio-Rad, Hercules, USA).

RETRACTED

### Statistical analyses

All experiments were done in triplicate. The results of multiple experiments are reported as means±SD. Statistical analyses were performed using SPSS 19.0 statistical software (USA). P values were calculated using one-way analysis of variance. P<0.05 was considered to be statistically significant.

## Results

### UVB induced HaCaT cell injury

Exposure of HaCaT cells to UVB decreased cell viability (Figure 1A) and increased apoptosis (Figure 1B) in a time-dependent manner. Western blot analysis for apoptosis (Figure 1C) also showed similar results, with increase in the expressions of pro-apoptotic proteins (Bax, cleaved caspase 3 and 9) and decrease in the expression of anti-apoptotic protein (Bcl-2).

**Figure 1.** UVB induced HaCaT cell injury; *A*, Cell viability assay revealed UVB inhibited HaCaT cell viability; *B*, Apoptosis assay revealed UVB promoted HaCaT cell apoptosis; *C*, Western blotting analysis revealed increased expression of Bax, decreased expression of Bcl-2, and activation of caspase-3 and caspase-9; *D*, ELISA results demonstrated that UVB promoted the expression of TNF-α; *E*, ELISA results demonstrated that UVB promoted the expression of IL-6; *F*, Western blotting analysis revealed overexpression of TNF-α and IL-6 in UVB-induced cells. Data are reported as means±SD. **P<0.01, ***P<0.001 compared to control (ANOVA). UVB: ultraviolet B; ELISA: enzyme-linked immunosorbent assay; TNF-α: tumor necrosis factor-α; IL-6: interleukin-6.

The results of ELISA showed significantly increased expressions of TNF-α (P<0.001, Figure 1D) and IL-6 (P<0.001, Figure 1E) in UVB-treated HaCaT cells compared to non-irradiated control cells. Similar results were obtained by western blotting analysis (Figure 1F). The results indicated that UVB induced cell inflammatory injury in HaCaT cells.

RETRACTED

### UVB up-regulated the expression of HOTAIR

The results of quantitative RT-PCR showed that HOTAIR was highly expressed at 16 h of UVB exposure (Figure 2). Therefore, subsequent experiments were conducted with a UVB treatment time of 16 h.

**Figure 2.** qRT-PCR was performed to evaluate the effect of UVB on HOTAIR and data revealed that UVB upregulated the expression of HOTAIR. Data are reported as means±SD. ***P<0.001, compared to control (0 UVB) (ANOVA). qRT-PCR: quantitative real-time polymerase chain reaction; UVB: ultraviolet B; HOTAIR: HOX antisense intergenic RNA.

### Effect of HOTAIR on UVB-induced cell injury

The results of RT-PCR (Figure 3A) showed significantly increased expression of HOTAIR in pc-HOTAIR group compared to pc-DNA3.1 (P<0.001), and significantly decreased expressions of HOTAIR in sh-HOTAIR#1 and #2 group compared to sh-NC (P<0.05 and P<0.01). We then measured the effects of altered expression of HOTAIR on cell viability, apoptosis, and pro-inflammatory cytokine concentration in UVB-treated cells. Overexpression of HOTAIR significantly decreased cell viability (P<0.05; Figure 3B), increased apoptosis (P<0.01; Figure 3C), inhibited Bcl-2 expression (P<0.01; Figure 3D), altered apoptosis-associated factors (Figure 3E), and increased the expressions of TNF-α (P<0.05; Figure 3F and H) and IL-6 (P<0.05; Figure 3G and H) compared with the pcDNA3.1 group in UVB-treated cells. In contrast, suppression of HOTAIR expression using sh-HOTAIR#1 and #2 significantly increased cell viability (both P<0.05; Figure 3B), decreased apoptosis (both P<0.05; Figure 3C), and increased Bcl-2 expression (P<0.05; Figure 3D). No significant difference was found between sh-HOTAIR#1 and #2 transfection group. Due to the higher transfection efficiency of sh-HOTAIR#2, it was used for subsequent studies. We also found that inhibiting HOTAIR expression decreased the expressions of Bax, cleaved caspase-3, and cleaved caspase-9 (Figure 3E). Inhibiting HOTAIR expression reduced TNF-α (P<0.05; Figure 3F and 3H) and IL-6 (P<0.01; Figure 3G and H) compared with sh-NC in UVB-treated cells. The results indicated that suppression of HOTAIR alleviated UVB-induced cell injury and overexpression of HOTAIR further promoted UVB-induced cell injury.

**Figure 3.** Effect of HOTAIR on UVB-induced cell injury; *A*, qRT-PCR revealed overexpression and suppression of HOTAIR in HaCaT cells after transfection assay; *B*, Cell viability assay revealed suppression of HOTAIR alleviated UVB-induced low cell viability and overexpression of HOTAIR further promoted UVB-induced inhibition of cell viability; *C*, Apoptosis assay revealed suppression of HOTAIR alleviated UVB-induced high cell apoptosis and overexpression of HOTAIR further promoted UVB-induced high cell apoptosis. *D*, qRT-PCR analysis showed that mRNA expression of Bcl-2 was increased after HOTAIR was silenced and decreased after HOTAIR was overexpressed. *E*, Western blotting analysis showed increased expression of Bax and decreased expression of Bcl-2 in HOTAIR overexpressed cells; *F*, ELISA results showed suppression of HOTAIR alleviated UVB-induced high expression of TNF-α and overexpression of HOTAIR further promoted UVB-induced high expression of TNF-α; *G*, ELISA results showed suppression of HOTAIR alleviated UVB-induced high expression of IL-6 and overexpression of HOTAIR further promoted UVB-induced high expression of IL-6; *H*, Western blotting analysis showed increased expression of TNF-α and IL-6 with HOTAIR overexpression. Data are reported as means±SD. *P<0.05; **P<0.01; ***P<0.001 (ANOVA). ns: P>0.05. UVB treatment time was 16 h. HOTAIR: HOX antisense intergenic RNA; UVB: ultraviolet B; qRT-PCR: quantitative real-time polymerase chain reaction; TNF-α: tumor necrosis factor-α; IL-6: interleukin-6.

RETRACTED

The effects of HOTAIR on HaCaT cells with no UVB treatment were also analyzed in this study (Supplementary Figure S1). Inhibiting HOTAIR increased cell viability, but had no significant effect on apoptosis or expression of pro-inflammatory factors. Enhancing HOTAIR expression inhibited viability, promoted apoptosis, and elevated expressions of TNF-α and IL-6. Thus, we speculated that HOTAIR might be an important regulator in HaCaT cells.

### HOTAIR promoted the expression of RNA-dependent protein kinase (PKR)

Quantitative RT-PCR was performed to evaluate the effect of HOTAIR on the expression of PKR (Figure 4A). Results showed that overexpression of HOTAIR significantly promoted the expression of PKR (P<0.01), while suppression of HOTAIR using sh-HOTAIR#1 and #2 decreased the expression of PKR (both P<0.05). Similar results were obtained by western blotting analysis (Figure 4B).

**Figure 4.** Effect of HOTAIR on PKR expression; *A*, qRT-PCR revealed overexpression of HOTAIR promoted the expression of PKR; *B*, Western blotting analysis revealed overexpression of HOTAIR promoted the expression of PKR. Data are reported as means±SD. *P<0.05; **P<0.01 (ANOVA). HOTAIR: HOX antisense intergenic RNA; PKR: RNA-dependent protein kinase; qRT-PCR: quantitative real-time polymerase chain reaction.

### Effect of PKR on UVB-induced cell injury

Next, we investigated the effect of PKR on UVB-induced cell injury. Designed si-PKR#1 and 2 were transfected into cells and it was found that PKR expressions in both mRNA and protein were inhibited (both P<0.01, Figure 5A and B). The full-length PKR sequences were constructed into pcDNA3.1 plasmids (pc-PKR), and, as expected, pc-PKR significantly increased the mRNA expression (P<0.01; Figure 5C) and protein expression (Figure 5D) of PKR. We then measured the effects of altered expression of PKR on cell viability and apoptosis in UVB-treated cells. Overexpression of PKR significantly decreased cell viability (P<0.05; Figure 5E) and increased apoptosis (P<0.01; Figure 5F and G), compared with pcDNA3.1 group in UVB-treated cells. In contrast, suppression of PKR expression significantly increased cell viability (P<0.05; Figure 5E) and decreased apoptosis (P<0.05; Figure 5F and G), compared with sh-NC in UVB-treated cells.

RETRACTED

**Figure 5.** Effect of PKR on UVB-induced cell injury; *A* qRT-PCR revealed downregulation of PKR in HaCaT cells; *B,* Western blotting analysis revealed downregulation of PKR in HaCaT cells; *C*, qRT-PCR revealed overexpression of PKR in HaCaT cells; *D*, Western blotting analysis revealed overexpression of PKR in HaCaT cells; *E*, Cell viability assay revealed overexpression of PKR promoted UVB-induced cell viability inhibition, and the effects were reduced by suppression of PKR; *F*, Apoptosis assay revealed overexpression of PKR promoted UVB-induced cell apoptosis, and the effects were reduced by suppression of PKR; *G*, Western blotting analysis revealed overexpression of PKR promoted UVB-induced alterations in apoptosis-associated factors, and the effects were reduced by suppression of PKR. Data are reported as means±SD. *P<0.05; **P<0.01 (ANOVA). UVB treatment time was 16 h. PKR: RNA-dependent protein kinase; UVB: ultraviolet B; qRT-PCR: quantitative real-time polymerase chain reaction.

### Effect of HOTAIR and PKR on UVB-induced cell injury

We then measured the effects of altered expressions of PKR and HOTAIR in combination on cell viability, apoptosis, and pro-inflammatory cytokine concentration in UVB-treated cells. For this, UVB-treated cells were transfected with pcDNA3.1+siNC, pc-HOTAIR+siNC, and pc-HOTAIR+si-PKR. As presented previously, overexpression of HOTAIR significantly decreased cell viability (P<0.05; Figure 6A), increased apoptosis (P<0.01; Figure 6B and C), and increased the concentrations and protein expression of TNF-α (P<0.05; Figure 6D and F) and IL-6 (P<0.05; Figure 6E and F) compared with pcDNA3.1 in UVB-treated cells. However, suppression of PKR expression reversed these effects by significantly increasing cell viability (P<0.01; Figure 6A), decreasing apoptosis (P<0.01; Figure 6B and C), and increasing the expressions of TNF-α (P<0.01; Figure 6D and F) and IL-6 (P<0.01; Figure 6E and F), compared with pc-HOTAIR in UVB-treated cells. These results suggested that overexpression of HOTAIR promoted UVB-induced cell injury by upregulation of PKR.

RETRACTED

**Figure 6.** Effect of HOTAIR and PKR on UVB-induced cell injury; *A*, Cell viability assay demonstrated overexpression of HOTAIR promoted UVB-induced cell viability inhibition by upregulation of PKR, and suppression of PKR reversed the results; *B,* Apoptosis assay showed overexpression of HOTAIR promoted UVB-induced cell apoptosis by upregulation of PKR, and suppression of PKR reversed the results; *C,* Western blotting analysis revealed overexpression of HOTAIR promoted the effects of UVB on apoptosis-related factors by upregulation of PKR, and suppression of PKR reversed the results; *D* and *E*, ELISA revealed overexpression of HOTAIR promoted UVB-induced high expression of TNF-α and IL-6 by upregulation of PKR, and suppression of PKR reversed the results; *F*, Western blotting analysis showed overexpression of HOTAIR promoted UVB-induced high expression of TNF-α and IL-6 by upregulation of PKR, and suppression of PKR reversed the results; *G*, Inhibiting expression of HOTAIR reversed the viability-inhibitory effect of PKR; *H*, Inhibiting expression of HOTAIR reversed the apoptosis-promoting effect of PKR; *I*, HOTAIR silence reversed the effects of PKR on apoptosis-related factors. Data are reported as means±SD. *P<0.05; **P<0.01 (ANOVA). UVB treatment time was 16 h. HOTAIR: HOX antisense intergenic RNA; PKR: RNA-dependent protein kinase; UVB: ultraviolet B; qRT-PCR: quantitative real-time polymerase chain reaction; TNF-α: tumor necrosis factor-α; IL-6: interleukin-6.

As described previously, PKR overexpression inhibited cell growth and promoted cell inflammation. These effects were also impaired by HOTAIR silence (Figure 6G, H, and I), which indicated that growth and inflammation injury of UVB-treated cells were affected by interaction between HOTAIR and PKR.

### Effect of PKR on PI3K/AKT and NF-κB signaling pathways

Lastly, we measured effects of PKR on PI3K/AKT and NF-κB signaling pathway-related proteins (PI3K, AKT, p-65, and IκBα) in UVB-treated cells using western blot (Figure 7A and B). Overexpression of PKR increased the expression of phosphorylated PI3K, AKT, p65, and IκBα, whereas suppression of PKR expression showed the opposite effects. These results suggested that overexpression of PKR activated PI3K/AKT and NF-κB pathways in UVB-injured HaCaT cells.

**Figure 7.** Western blotting analysis of PKR on PI3K/AKT and NF-κB signaling pathways, which suggested that overexpression of PKR activated *A*, PI3K/AKT pathway and *B*, NF-κB pathway. UVB treatment time was 16 h. UVB: ultraviolet B; PKR: RNA-dependent protein kinase; PI3K: phosphatidylinositol-3 kinase.

RETRACTED

## Discussion

In the present study, we explored the effects of HOTAIR on UVB-induced keratinocyte injury. The results showed that UVB induced HaCaT cell injury and upregulated the expression of HOTAIR. Overexpression of HOTAIR further promoted the UVB-induced cell injury and suppression of HOTAIR reduced the cell damage. Further studies showed that HOTAIR upregulated the expression of PKR, activating the PI3K/AKT and NF-κB pathway.

Repeated UVB exposure results in damage to skin cells and induction of carcinogenesis (15,16), which requires the rapid removal of irreparably damaged cells after exposure to UV irradiation and condemned to cell apoptosis (17). It is important to maintain the balance of proliferation, stratification, differentiation, and apoptosis of skin cells for epidermal homeostasis (18); DNA damage repair and induction of apoptosis are main cellular mechanisms for this balance.

As an important epigenetic regulation mechanism of gene expression under environmental stress, lncRNAs have been found to play important roles in environmental response (19). Several techniques have been applied to study the molecular mechanisms underlying UVB-induced photo damage and skin carcinogenesis, and lncRNAs have been shown to be involved in this process (8). However, the specific functions of HOTAIR and the underlying mechanisms are still unknown in UVB-induced skin injury. The importance of lncRNAs has been implicated in many different contexts. HOTAIR interacts with Polycomb Repressive Complex 2 (PRC2) and is necessary for PRC2 occupancy and histone H3 lysine-27 trimethylation of different genes in different chromosomes. PRC2 is a histone methyltransferase that implements epigenetic silencing during different processes, including cancer development (20).

Our study revealed that overexpression of HOTAIR promoted UVB-induced apoptosis and inflammatory injury by up-regulation of PKR in keratinocytes. Several studies have shown antiviral defense mechanism through PKR in keratinocytes (21). Also, the association of HOTAIR and PKR has been demonstrated in several different cancers (22 [Bibr B23]–24). However, no study has evaluated the association of HOTAIR and PKR in UVB-induced cell injury. Our study showed that overexpression of HOTAIR significantly promoted the expression of PKR, while suppression of HOTAIR inhibited the expression of PKR.

Several protein kinases are involved in the UV-induced signal transduction (25). To our knowledge, this is the first study that demonstrated the role of PKR in UVB-induced skin injury. However, the role of PKR in activation of inflammasome has been confirmed. Lu et al. (13) demonstrated that PKR activity was integral to assembly and activation of inflammasome and that it mediated inflammatory response by activating caspase-1, cleavage IL-1β, and releasing HMGB1. PKR was involved in inflammation and immune dysfunction through regulating mitogen-activated protein kinases (MAPKs), interferon regulatory factor 3 (IRF3), NF-κB, apoptosis, and autophagy pathways (26). These studies indicated the pro-inflammation effect of PKR, which were consistent with our study.

RETRACTED

There are several pathways involved in UVB-induced skin injury as solar UVB radiation induces erythema, sunburn, hyperplasia, proliferation, inflammation, oxidative stress, DNA damage, p53 mutations, immunosuppression, and alterations in PI3K/AKT and NF-κB cell survival signaling pathways eventually leading to skin cancer (27 [Bibr B28] [Bibr B29] [Bibr B30]–31). UVB-induced inflammatory responses include increased production of pro-inflammatory cytokines such as TNFα, IL-1β, and IL-6 (32,33). UVB radiation activates PI3K/AKT pathway in cultured cells as well as in both mouse and human skin (34 [Bibr B35]–36). In UVB-exposed skin, PI3K/AKT signaling increases the survival response of keratinocytes and facilitates tumorigenesis (37). Also, NF-κB regulates production of inflammatory mediators and induces transcription of pro-inflammatory genes. NF-κB also contributes to the regulation of cell proliferation and survival. Previous studies have shown that UVB radiation activates NF-κB signaling in keratinocytes and mouse skin (38 [Bibr B39]–40). Our study showed that overexpression of PKR activated PI3K/AKT and NF-κB pathways.

In conclusion, our study findings suggested that overexpression of HOTAIR promoted UVB-induced cell injury in HaCaT cells. Overexpression of HOTAIR upregulated the expression of PKR, leading to the activation of PI3K/AKT and NF-κB pathways. These results indicated that HOTAIR promoted UVB-induced apoptosis and inflammatory injury by up-regulation of PKR in keratinocytes.

## Supplementary material

Click here to view [pdf].
